This article has been retracted.

# Emergency Medicine with Advanced Surgery Protocols: A Review

**DOI:** 10.1155/2022/3513250

**Published:** 2022-09-26

**Authors:** Hilla Mills, Ronald Acquah, Nova Tang, Luke Cheung, Susanne Klenk, Ronald Glassen, Magali Pirson, Alain Albert, Duong Trinh Hoang, Thang Nguyen Van

**Affiliations:** ^1^Clinical Center of Vojvodina, Novi Sad, Serbia; ^2^Clinical Analysis Lab, Center of Bio-Medicine, Hanoi, Vietnam; ^3^RD Lab, The Hospital Institute for Herbal Research, 50200 Toluca, MEX, Mexico; ^4^Research Institution of Clinical Biomedicine, Hospital University Medical Centre, 89000 Ulm, Germany; ^5^Industrial Research Group, International College of Science and Technology, Route de Lennik 800, CP 590, 1070 Brussels, Belgium

## Abstract

One of the most burning issues in health system is the concern of handling patients that requires emergency surgery. Emergency general surgery is done on both traumatic and nontraumatic acute disorders. Severe traumatic injury and bleeding is one of the causing agents for high mortality rate globally. Another group of patients that are in need of emergency surgery are those with heart failure, and in this particular paper, we analyzed emergency medicine with advanced surgery protocols focusing on gastric cancer, cardiac surgery, and bleeding as well as coagulopathy following traumatic injury.

## 1. Introduction

Emergency medicine is a field of practice that utilizes knowledge and skills required for the injury affecting patients. The set of skills involve prevention, diagnosis, and management of sensitive illness [1]. Emergency medicine deals with patients that are in a critical condition, which could either be seriously injured or seriously ill patients who need emergency attention [2]. Therefore, emergency medicine is mostly taken care of or given in hospitals and clinics where the vital care needed is readily available. David et al. made it clear that emergency medicine is practiced differently around the different parts of the world, since people define emergency medicine differently [2–4].

This difference that arises in the definition of emergency medicine arises because of the ailments that each nation has such that it would be of no use to apply the same understanding of emergency medicine. The population at large has also their duty to give full support to the advancement of emergency medical services and prehospital development, aid in disaster relief as well fight to prevent accidents, and recognize and advance academic emergency medicine. Once more, this has been amply noted in emergency medicine studies published in India, Japan, and some parts of Europe [4]. In this particular paper, we discussed the importance of emergency medicine focusing on the advanced surgery protocols in cardiac surgery, gastric cancer, and bleeding as well as coagulopathy following traumatic injury.

## 2. Major Bleeding and Coagulopathy

It takes one to have a very deep understanding of the biology behind the reaction to trauma as well to be able to manage trauma patients with severe injuries. This has led to modifications of known treatment of trauma combined with injuries such that there are recent advances in clinical and basic science research towards the treatment of patients with bleeding trauma [5]. In about 10 cases of bleeding trauma patients, 3 cases exhibit indications of coagulopathy and the situation where patients would bleed following emergency medicine operations. The bleeding is deemed to be one of the causes of avoidable death among injured patients [6–9]. These patients with posttraumatic bleeding are said to be in a very critical condition as they can also die from multiple organ failure [10]. Thrombin-thrombomodulin complex generation mainly is a factor that has shown to cause early acute coagulopathy which is linked to traumatic injury [11]. Coagulation disease can be worsened by factors like therapeutic and environmental factors that cause acidaemia, hypothermia, dilution, hypoperfusion, and consumption of coagulation [12], and trauma causes brain injury as shown in Figure 1.

### 2.1. Advanced Surgery for Bleeding

In the situation that it occurs that a patient has been severely injured, and there is hemorrhagic shock, bleeding, and coagulopathy, it is advised that the patient undergoes damage-control surgery. For patients suffering from hypothermia, acidosis, and anatomical injuries that are inaccessible, simultaneous significant harm outside the abdomen may also go through a damage-control surgery [13]. It is believed that if a critically injured person does not receive bleeding management and appropriate resuscitation, blood transfusion has low chances of surviving.

This is more dangerous when the patient is suffering from a number of penetrating injuries and uncontrolled bleeding. The other group of patients at risk of losing their lives is those who have serious abdominal injuries and pelvic fractures that will be bleeding and retroperitoneal arteries. The methods of limiting hemorrhage, laparotomies, and delaying final surgical repair until coagulation has been established were all described by Morris et al. in 1983 [14]. The strategy is now known as damage control [15–17]. This method is now being employed on patients who have sustained a serious abdominal injury and to patients in need of adjunctive angioembolization. Patients suffering from traumatic amputation of a limb, severe stomach injuries, and injuries as soon as feasible can also be treated with damage control surgery. Improvements in the damage-control surgery include a temperature 34°C, pH 7.2 when carrying out the surgery [18, 19].

Additionally, an accelerated resuscitative laparotomy is performed as part of damage-control surgery for the abdomen in order to reduce bleeding, restore blood flow when necessary, and prevent contamination. This is now being done soon so as not to waste time on conventional organ repairs as these can be done at a later stage. The abdomen is packed; packing may allow to compress ruptures in the liver and to provide direct pressure to the sites where bleeding will be taking place. Rebleeding is avoided by removing the removal of packs for about 48 hours. In this part, the patient's temperature control is also very important. In the emergency operation, the patient's hypothermia reduces the productivity of the damaged body, and a large amount of heat energy dissipates during the operation. However, most surgeons tend to ignore the links of operating room warming, patient's body heat preservation, infusion fluid and irrigation fluid heating, and so on. Therefore, hypothermia generally exists in severely injured patients. In this case, the patient will suffer from systemic cell metabolism disorder, arrhythmia, reduction of cardiac output, prompting oxygen dissociation curve to move to the left and reducing the release of oxygen between tissues, etc., thus affecting the coagulation function, and the death rate of the patient will increase from 40% to 100%.

The next step of damage-control surgery would be intensive care, which is mainly about rewarming, coagulopathy correction, acid-base balance, and haemodynamic optimization. The final surgical repair, which is the third step, is normally carried out when the rewarming, coagulopathy correction, acid-base balance, and haemodynamic optimization have been reached [16, 17]. The surgical procedure's less harsh nature and brief duration are intended to lessen secondary procedure-related trauma.

### 2.2. Reamed Nailing

Long bone fractures are usually dealt with using reamed nailing technique. The method is known to be the standard method that can be safely used in treatment of long bone fractures. It has been a problem with reaming since it would lead to the undesired effects like heat generation, issues with reamer flutes, and fat embolization [18]; however, the technique has been improved such that to overcome fat intravasation caused by increased intramedullary pressure, and the reamed irrigator aspirator (RIA) device was developed. The device has shown to lessen the side effects of reaming as it minimizes remobilization [19, 20], and currently, this device is being used, especially in bone graft [21]. A device that cuts like RIA needs accurate cutting in the medullary canal compared to the usual reamers; therefore, another complex version of RIA device has been invented which overcomes the drawback of the cutting-head size of the firstly developed RIA device which is small and with issues also in connection between the drive shaft and the cutting head.

### 2.3. Definitive Surgery

Safe fracture fixation in badly injured people normally experience inflammatory changes especially in the neutrophil level [22]. There has been a technique that was developed which detects if the neutrophils are present in the body of a badly injured person [23]. This is of importance as it will contribute to make a decision that inflammatory and soft tissue injury-induced alterations can be returned back to normal by a surgery. Cardiac function was revealed to be more damaged when RIA 1 is used but showed to be successful when RIA 2 was used [24, 25]. This information is important as it ensures safe definitive surgery and also reinforces the importance of patient assessment to achieve the goal of safe definitive surgery [26]. Therefore, it is encouraged to use many factors together as they have shown to be helpful in surgery, and these advances for surgeries will be helpful in coming up with successful surgeries [27].

## 3. Gastric Cancer

Gastric cancer is considered to be in the top 3 of fatal cancers. Many death cases have been recorded to have been caused by gastric cancer [28]. The disease has been treated using the *H. pylori* treatment; however, the cases keep rising and the treatment has shown not be effective. The disease requires screening but the screening is very expensive; thus, many people only realize that they are suffering from gastric cancer when it becomes severe. Therefore, advanced treatment of gastric cancer has been invented which includes advanced minimally invasive surgical procedures. Thus, in recent years, the incidence and mortality of gastric cancer in many countries with high incidence of gastric cancer, including Japan, have shown a decreasing trend in different degrees. The reasons are mainly related to the decrease of Helicobacter pylori infection rate, the decrease of salt intake, the increase of fresh vegetable and fruit intake, and the radical endoscopic treatment after gastric cancer screening and early detection [29].

### 3.1. Advances in Gastric Cancer Treatment

Complete surgical resection has become the gastric cancer treatment such that total gastrectomy and subtotal gastrectomy are the popular methods that are now being used in treating gastric cancer. Gastrectomy procedure goes along in combination with lymphadenectomy to achieve oncologic resection and staging of gastric cancer and D3 (perigastric, eliac axis, and para-aortic lymph node stations) lymphadenectomies. Studies have revealed that patients have more survival rate when they are treated with this combination compared to when treated with lymphadenectomy alone [30].

Gastrectomy, in the treatment of stomach cancer, has become the choice of many as it comes along with many benefits such as reduced blood loss, lower morbidity, and a quicker recovery of bowel function compared to chemotherapy. The survival rates for chemotherapy and radiation have been shown to much lower compared to those for gastrectomy [31]. Cytoreductive surgery and heated intraperitoneal chemotherapy are also under investigation to treat peritoneal illness. Studies have revealed that patients with advanced gastric cancer who underwent heated intraperitoneal chemotherapy after cytoreductive surgery recovered [32].

## 4. Cardiac Surgery

Despite its high cost, cardiac surgery is the only accepted standard therapy for the treatment of heart disease on a global scale. Percutaneous and surgical treatments for coronary artery disease as well as surgical adjuvant such cardiac imaging and blood conservation have all benefited from advancements in cardiac surgery.

### 4.1. Coronary Surgery vs. Percutaneous Coronary Intervention

For single vessel disease, percutaneous coronary intervention was done; however, coronary stenting and surgical methods were not frequently employed. Coronary artery reperfusion therapy has significantly improved the clinical prognosis of patients with acute myocardial infarction (AMI). However, coronary angiography confirmed that in some successful emergency percutaneous coronary intervention (PCI), the myocardial tissue on the verge of necrosis or severe ischemia did not fully and effectively restore blood perfusion, which was related to no-reflow phenomenon. The incidence of no-reflow after reperfusion in acute myocardial infarction is 10%~30%. No-reflow greatly reduces the clinical benefits of emergency PCI. Compared with patients with normal forward coronary blood flow, these patients often have cardiac insufficiency and angina pectoris after infarction. And bypass surgery is a far more intrusive alternative to coronary stenting for revascularization. Stents are employed because they have lower rates of restenosis than balloon angioplasty alone, and they also play a crucial role in the management of angioplasty-related problems [33].

### 4.2. Pump Surgery

During coronary artery bypass surgery, cardiopulmonary bypass can either be employed (known as “on-pump”) or not used at all (known as “off-pump”). Up until recently, the majority of surgeons used on-pump procedures since it was thought that off-pump surgery reduced patients' risk of stroke. Off-pump surgery has been shown to perform better than on-pump surgery by reducing postoperative atrial fibrillation, the need for transfusions and inotropes, ventilation times, hospital stay length, and cost [34]. Numerous researches have also looked into the issue of patients receiving fewer grafts in off-pump groups [35].  Table 1 shows different ways of performing coronary surgery.

### 4.3. Atrial Fibrillation Surgery

With a high mortality rate and increased risk of stroke, postoperative atrial fibrillation affects roughly 38% of patients having mitral valve surgery. But for patients having mitral surgery, the Maze III procedure is the gold standard for treating atrial fibrillation currently: over 85% of patients who undergo the standard Maze surgery are cured of atrial fibrillation [36], but because to its complexity, the Maze III is only performed by a small number of surgeons. Though thoracoscopic and minimally invasive approaches have been made easier by new ablation technologies like radiofrequency, microwave, and cryotherapy, the indications for surgical treatment of atrial fibrillation will likely continue to be restricted to those with concurrent cardiac surgical pathology needing surgery.

### 4.4. Preservation of Blood

According to data from the National Blood Service, cardiac surgery uses a lot of blood. Therefore, blood conservation measures have been put in place. These tactics lead to postoperative bleeding and transfusions as well as a decreased supply of blood components. Both tranexamic acid and aprotinin are antifibrinolytics that, when used after heart surgery instead of a placebo, significantly reduce the need for blood transfusions and reoperations due to bleeding [37]. In this meta-analysis, neither medication was discovered to be linked to noticeably higher rates of adverse events. Blood is drawn from the surgical site or postoperative drains by cell salvage systems, which then heparinize, cleanse, and generate concentrated red blood cells that can be given back to the patient. According to calculations, the likelihood of needing a blood transfusion is nearly eliminated with washed cell salvage. Variations in transfusion thresholds were a substantial source of variability in the research included in both meta-analyses. There is no longer a need for placebo-controlled trials of either approach in cardiac surgery, according to both of these meta-analyses. Research that identify the risk-benefits of allogeneic blood transfusion in cardiac surgery as well as studies that determine the haematocrit that maximizes coronary anastomotic patency and myocardial oxygen delivery are presently required [38].

### 4.5. Heart Failure Surgery

In carefully choosing patients with ejection fractions under 20 percent, enough reserves of dormant myocardium, and acceptable coronary anatomy, it has been demonstrated that cardiac artery bypass grafting provides superior outcomes to cardiac transplantation. Relative contraindications to cardiac artery bypass grafting include right ventricular failure and increased pulmonary artery pressure. Operative mortality in this high-risk category has been decreased to 7% thanks to careful patient selection and temporary mechanical assistance, and the 5-year survival rate has reached approximately 80% [39]. In cardiac failure, mitral regurgitation frequently occurs. Due to the high rate of surgical mortality in the 1980s, it was thought that the elimination of the low resistance regurgitant channel would inevitably result in a postoperative decline in left ventricular function. Hospital mortality in one series was as low as 2% due to better understanding of the necessity to protect the subvalvular apparatus, correct and prevent annular dilatation, and enhance mitral valve repair procedures [39]. The Thoratec HeartMate left ventricular assist device was given approval by the US Food and Drug Administration in 2003 for long-term treatment of patients with end-stage heart failure. Data showing that the placement of a left ventricular assist device reduced 1-year mortality by a third relative to medical care were used to support approval [39]. In many patients, early bleeding and late infection continue to be issues.

## 5. Conclusion

At present, the professional differentiation of emergency department is getting finer and finer, and the theoretical knowledge and clinical skills of many specialists are becoming more and more specialized, which leads to the fact that although emergency department is a complete department, it has to shoulder more responsibilities, and many chronic diseases often exist at the same time in different regions and different ages. However, some chronic diseases are acute, or new acute diseases are acquired on the basis of many chronic diseases. At this time, the diseases of various systems cross each other and occur in one patient, which is by no means something that a single specialist can solve. Therefore, it is necessary for emergency doctors to comprehensively evaluate and analyze the pathophysiological state of patients, so as to give targeted treatment to patients, so that patients can get the most scientific treatment in the golden time. And there have been numerous advances in surgical methods in cardiac surgery. Future research may concentrate on stem-cell-based therapy and biotechnology, particularly in relation to surgery for heart failure, while the proper management of trauma patients with massive bleeding and coagulopathy continues to be a major challenge in routine clinical practice, and the management of gastric cancer is a challenge requiring a multidisciplinary approach for optimal treatment, so future research on gastric cancer may concentrate on next-generation genomic analysis.

## Figures and Tables

**Figure 1:** Conditions that are associated with trauma and traumatic coagulopathy shown in a series of steps.

**Table 1:** Invasive techniques in coronary artery bypass grafting.

Technique	Description
Off-pump coronary artery bypass (OPCAB)	Any coronary artery bypass surgery carried out without cardiopulmonary bypass
Minimally invasive direct coronary artery bypass (MIDCAB)	Surgery performed off-pump through a small thoracotomy under direct vision
Endoscopically assisted atraumatic coronary artery bypass (Endo-ACAB)	Internal mammary artery harvested endoscopically, coronary anastomosis performed off-pump through a minithoracotomy under direct vision
Totally endoscopic coronary artery bypass (TECAB)	Surgery performed off-pump entirely endoscopically with robotic assistance
Hybrid	MIDCAB, Endo-ACAB, or TECAB with elective percutaneous coronary stenting of additional stenoses

## Data Availability

The data used to support the findings of this study are included within the article.
